This article has been retracted.

# Eagle Syndrome: A Rare Cause of Stroke in a Young Patient

**DOI:** 10.7759/cureus.21102

**Published:** 2022-01-11

**Authors:** Hussain A Alobaidi, Ali A Alfaran, Hawa H Algazwi, Fatimah I Alkhater, Hussain M Alshooalah, Abdulrahman K Alanzi, Ibrahim A Almindil, Abdullah K Alqasim, Aisha A Faqeeh, Amani A Almutairi, Ghaida H Alnaqa, Najla H Alnaqa, Renad M Alasmari, Razan M Almashouf, Faisal Al-Hawaj

**Affiliations:** 1 Medicine, Misr University for Science and Technology, 6th of October, EGY; 2 Dentistry, Imam Abdulrahman Bin Faisal University, Dammam, SAU; 3 Medicine, Almaarefa University, Riyadh, SAU; 4 Medicine, King Abdulaziz University, Jeddah, SAU; 5 Dentistry, King Saud bin Abdulaziz University for Health Sciences, Riyadh, SAU; 6 Dentistry, Riyadh Elm University, Riyadh, SAU; 7 Emergency Medicine, Imam Abdulrahman Bin Faisal University, Dammam, SAU

**Keywords:** str, temporomandibular disorder, neck pain, case report, eagle's syndrome

## Abstract

Stroke is a common acute neurological injury that may develop due to arterial thrombosis or hemorrhage. However, it is uncommon in the young population. The etiologies of stroke in young patients are different compared with those for the elderly population. They include various non-atherosclerotic angiopathies, hematological conditions, and inflammatory disorders. We report the case of a 26-year-old man who presented to the emergency department because he noticed that his right hand had become clumsy. He first noticed this symptom five days before his presentation, but he noticed that his symptom had improved significantly since it began. He reported that he had episodes of neck pain and pain around the ear. He visited the family physician clinic several times for this complaint and was diagnosed as having a temporomandibular joint disorder. Neurological examination revealed decreased muscle strength in the right upper limb with a power of 4/5 along with a sensory deficit. The coordination was intact. No gait ataxia was noted. Considering the patient’s age, the initial diagnosis was a demyelinating disorder such as multiple sclerosis. The patient underwent magnetic resonance imaging of the brain. It demonstrated an increased signal intensity in the territory of the left middle cerebral artery representing a left-sided infarction. Subsequently, the patient underwent computed tomography angiography of the head to rule out any structural malformation. The scan showed the presence of an elongated styloid process that appeared in close proximity to the neck vasculature. These radiological findings are consistent with Eagle syndrome. The patient underwent surgical resection of the styloid process. Eagle syndrome is a rare clinical condition that may have a myriad of clinical presentations. A high index of suspicion for this condition is vital to reach the diagnosis. Physicians should keep this condition in the differential diagnosis of stroke in the young population with no risk factors.

## Introduction

Stroke is an acute neurological injury that may develop due to thrombosis or hemorrhage. It is a common condition worldwide. However, stroke in the young population is uncommon and is a major cause of long-term morbidity. The etiologies of stroke in young adults differ from the classic risk factors of stroke in the elderly population [1]. These uncommon pathologies include non-atherosclerotic angiopathies such as cervicocephalic arterial dissection, fibromuscular dysplasia, and moyamoya disease. Furthermore, the hematological conditions are a very important predisposing factor for stroke in the young population [1]. Such conditions include inherited and acquired thrombophilia disorders, such as antiphospholipid syndrome and sickle cell disease. Inflammatory and infectious etiologies are also important and include different vasculitis disorders, such as Behçet disease [1]. Here, we present the case of a young healthy man with stroke as a manifestation of Eagle syndrome, an unusual cause of stroke in the young population. Eagle syndrome is an underrecognized clinical condition with a myriad of clinical manifestations related to the presence of elongated styloid processes [2].

## Case presentation

A 26-year-old man presented to the emergency department because he noticed that his right hand had become clumsy. He first noticed this symptom five days before his presentation, but he noticed that his symptom had improved significantly since it began. The weakness was associated with numbness in his right arm and hand. His symptoms developed suddenly while he was playing football. It was the first time for him to experience such symptoms. There was no history of visual disturbances, difficulty in speaking, gait disturbances, headache, or loss of consciousness.

The patient was otherwise healthy and did not have any history of hypertension, dyslipidemia, or diabetes mellitus. He reported that he had episodes of neck pain and pain around the ear. He visited the family physician clinic several times for this complaint and was diagnosed as having a temporomandibular joint disorder. He was prescribed naproxen 500 mg and local diclofenac gel. These episodes occurred around once every month and had spontaneous resolution with the symptomatic treatment. He had no history of previous surgeries. He maintained a healthy lifestyle and never smoked or used alcohol. He actively played sports and family history was unremarkable for sudden cardiac death.

On examination, he was fully oriented to time, place, and person. The vital signs did not show any abnormalities. Neurological examination revealed decreased muscle strength in the right upper limb with a power of 4/5 along with a sensory deficit. The coordination was intact. No gait ataxia was noted. Other systems showed normal physical examination findings. The laboratory findings, which included basic hematological and metabolic parameters, were normal. They revealed a hemoglobin level of 13.4 g/dL, leukocyte count of 8,500/μL, and platelet count of 380,000/μL. The electrolyte level included a sodium level of 135 mEq/L, potassium level of 4.1 mEq/L, and chloride level of 102 mEq/L. The albumin, bilirubin, and transaminases levels were within the normal reference range.

Considering the patient’s age, the initial diagnosis was a demyelinating disorder such as multiple sclerosis. The patient underwent magnetic resonance imaging of the brain. It demonstrated an increased signal intensity in the territory of the left middle cerebral artery representing a left-sided infarction (Figure 1). This finding of stroke was very unusual. Subsequently, the patient underwent computed tomography angiography of the head to rule out any structural malformation. The scan showed the presence of an elongated styloid process that appeared in close proximity to the neck vasculature (Figures 2, 3). These radiological findings are consistent with Eagle syndrome.

**Figure 1:** The MR image shows increased signal intensity in the left MCA territory representing stroke MR: magnetic resonance; MCA: middle cerebral artery

**Figure 2:** The CT image shows a prominent styloid process (arrows) in close proximity to vascular structures CT: computed tomography

**Figure 3:** CT angiography shows the elongated styloid processed (arrows) in close proximity to the carotid artery CT: computed tomography

The diagnosis was fully explained to the patient. The treatment options were discussed. Considering the serious complication that the patient had developed, surgical excision was advised. The patient underwent excision of the styloid process using the lateral approach. The operation was uneventful for complications and the patient was followed up for three years. He reported resolution of this frequent neck pain and had no active complaints.

## Discussion

We reported the case of Eagle syndrome in an otherwise healthy young man who presented with an ischemic stroke involving the left middle cerebral artery. Eagle syndrome is a rare idiopathic clinical condition that is associated with the elongated styloid process [3-5]. It has a myriad of clinical symptoms that classically include neck pain [2]. In the present case, the patient reported a previous history of neck pain that was misdiagnosed as a temporomandibular joint disorder.

The prevalence of Eagle syndrome varies significantly in the available literature [2]. Much of this variation is related to the difference in the cut-off point in the normal length of the styloid process. Some report that the abnormal length of the styloid process is more than 4 cm [4]. With this cut-off, the incidence of elongated styloid process was 4% [4-6]. However, not all patients with elongated styloid processes are symptomatic [2].

The clinical presentations of Eagle syndrome may include symptoms related to the compression of the internal carotid artery, as in the present case, and may present with syncope and ischemic stroke [2,7]. The first description of Eagle syndrome included two distinct groups of clinical syndromes. The classic syndrome includes neck pain, difficulty in swallowing, and globus sensation. The other described syndrome included compression of the carotid artery and visual disturbances and syncope [4,6].

A high index of clinical suspicion is very important to reach the diagnosis of Eagle syndrome. Plain and panoramic radiographs can suggest the diagnosis [3]. In the present case, the diagnosis was easily made by computed tomography scans. Furthermore, computed tomography angiography is essential to provide details about the carotid flow [4,8]. Eagle syndrome can be managed conservatively or surgically. The conservative management includes analgesics or local injections of anesthetics [3,6]. The surgical management can be performed by intra-oral or cervical approach [2,9]. In the present case, the cervical approach was performed as the treating surgeon was more familiar with this approach.

## Conclusions

Eagle syndrome is a rare clinical condition that may have a myriad of clinical presentations. A high index of suspicion for this condition is vital to reach the diagnosis. The diagnosis can be made by demonstrating an elongated styloid process in the computed tomography scan. Physicians should keep this condition in the differential diagnosis of stroke in the young population with no risk factors.
